RETRACTED

# Analysis on the Reform and Development of Physical Education Services in the Context of 5G Connected Communication

**DOI:** 10.1155/2022/5874248

**Published:** 2022-06-29

**Authors:** Li Wang, Dangyan Yan, Yanhong Zhang, Yuan Wen

**Affiliations:** ^1^Hebei Institute of Physical Education, Shijiazhuang 050041, China; ^2^College of Physical Education, Xingtai University, Xingtai 054001, China; ^3^Nanchang Institute of Technology, Nanchang 33108, China

## Abstract

With the continuous growth of science and technology, mankind has entered the fifth-generation (5G) era. In this background, the development of many fields will face great opportunities and challenges, including the field of physical education (PE). The traditional teaching mode, method, and contents of PE are difficult to adapt to the development needs of the 5G era. Therefore, it is of great significance to study the PE teaching reform in the era of “5G education.” Moreover, integrating 5G technology and PE may benefit students, educators, and the entire PE system. This study offers an in-depth investigation of the reforms and development of PE services under the background 5G interconnected communications. The reforms of PE and services are examined using the most up-to-date 5G technologies. Four 5G methodologies which include model-based practice (MBP), virtual reality (VR), the Internet of Things (IoT), and artificial intelligence (AI) are analyzed, and for the comparative study, performance indicators such as cost reduction, energy efficiency, and security level are measured. When compared to other strategies, IoT-based physical education is found to be more efficient in terms of these parameters. The 5G-driven PE will provide students with objective, fair, and diversified education, and adaptive learning services to promote the overall development of students.

## 1. Introduction

Physical education works to enhance students' physical experiences and abilities, as well as their overall well-being and ability to participate in a variety of physical activities. Physical education (PE) is typically characterized as a program that organizes sports and physical activity [1]. All of these activities contribute to a critical knowledge of the concept of PE. The PE focuses on physical fitness and the capacity to perform and enjoy physical activity. It enhances students' psychological and social capacities, as well as their physical, social, emotional, and psychological development. An effective study in PE is based on instruction, student, emotional health and trainers, quality education, and a student assessment [2].

In the application of 5G technologies, the development of high-quality PE teaching resources is an important requirement. The 5G communication not only increases students' access to the learning resources but also provides teachers with more ways to spread knowledge [3]. The traditional teaching mode has gradually been unable to meet the learning needs of students. In the 5G era, the time and space for students to acquire knowledge are no longer limited and the way for students to acquire knowledge is no longer only depending on the teacher but can learn and communicate through the network [4].

RETRACTED

Physical activity development in educational institutes employing environments and resources is currently ineffective [5]. The present management of physical activity and extracurricular activities is insufficient to meet the genuine demands of the student. Physical activities at educational institutions are generally isolated and analytically ineffective. The modern PE system is based on modern information technologies, IoT, and 5G communication networks [6]. Its core is students' training and PE, the provision of technical strategies, and the particular qualities of physical activities. The 5G communication networks and Internet of Things (IoT) can provide various opportunities to improve the education and training of PE [7]. Combining multiple applications of 5G communications with artificial intelligence, IoT data, and wearable physical analytics can precisely monitor each student's physical condition [8]. As part of the 5G and IoT association, cloud computing stores data from IoT devices in the cloud. In the cloud, PE resources can be kept on a centralized server that can be accessed anytime needed. IoT and 5G provide a convenient way to transmit and store that data. Infrastructures based on Internet cloud computing enable IoT to make sense of the vast quantity of data created. If student users use more or less storage, they may do it without any concern. As the volume of data created grows, they can simply scale up their storage and pay only for what they need with Internet cloud computing [9].

The conventional teaching mode of PE is hard to adapt to the development needs of 5G communication. Consequently, the application of PE teaching reform under the background of 5G and IoT is of great significance. In addition, the combination of 5G technology and PE may benefit students, teachers, and the entire PE system. In this context, this study offers an in-depth investigation of the reforms and development of PE services under the background of 5G interconnected communications. The reforms of PE and services are examined using the most up-to-date 5G technologies.

The rest of the manuscript is organized as follows: Section 2 provides a detailed description of the related works. In section 3, different existing technologies are discussed and analyzed.  Section 4 illustrates different results and provides a comparison of the different 5G technologies in promoting PE. Finally, the conclusion is given in section 5.

RETRACTED

## 2. Related Work

A student who participates in physical activities both in and out of school should have the abilities and confidence to engage in a variety of activities. With the support of a high-quality PE program that includes technology, all children may enjoy and achieve diverse physical activities. This section summarizes the complete literature review and highlights the most important studies on 5G and IoT PE monitoring and training. The 5G network services can improve communication performance and provide the best trade for linked IoT devices. Zhang [10] established an intelligent control technique for sports players' training development based on comprehensive data analysis. The intelligent control algorithm of sports athletes' training intensity was enhanced, and the operational efficacy of the intelligent control model of sports athletes' training intensity was secured, thanks to the development of the assessment system. The energy of the model was tested using simulations, and the results show that most models are successful. The intelligent model of athletes' training progress is advantageous for our study expansion in terms of analysis. The author in [11] developed a computing platform with optical fog nodes in the edge cloud middleware which offers an environment for a 5G network with ultra-fast equipment. The major objective of this system was to construct an optical fog node to be incorporated into the 5G system architecture for protective services applications by utilizing the computational power of optical resources. The author in [12] examined the 5G and AI data to find patterns and make sense of it so that end devices may take action. Moreover, they also explained the concepts of 5G and IoT technologies, as well as IoT-based 5G involved in the production, and then examined the problems and applicable solutions. To better understand the key function of the 5G mobile network, Hopkins et al. [13] first examined the practical importance of building a mobile communication network's main performance index scheme. Secondly, the performance standards of mobile communications are addressed in six different application scenes. Finally, the wireless transmission system's main performance index system was built. Jalal et al. [14] proposed the physical activity recognition system based on different sensors to detect physical activities from continuous sequences. Various sensors were deployed to record physical activities such as postures and actions, allowing sports individuals to get effective and timely care. Because the upcoming 5G network is projected to transform communication, IoT should be a major consideration in its design and standards. The author in [15] proposed that manufacturing smart solutions are enhanced by unique program applications such as mobile broadband (eMBB), massive machine-type communication (mMTC), ultra-reliable and low-latency communication (URLLC), and narrowband IoT (NB-IoT). The author in [16] offered Aerosmith, a new design framework for autonomously edge resource organization that includes small cell inclusion and topological management, and discussed the issues that the 5G mobile communications network faces, which include growing mobile data volumes, linking mass endpoints whenever and anywhere, spectrum scarcity, green environmental conservation, and clean energy. Casey et al. [17] created a planning model to estimate the necessary computation, memory, and wireless capabilities and used the number of values like net present value, internal rate of return, and estimated payback duration to evaluate the profitability of a possible investment in 5devices for immersion video services, taking into consideration dynamic elements like service penetration and pricing development. From the standpoint of 5G, this research investigated the use of virtual reality technology (VRT) in PE. In this study, different state-of-the-art technologies are examined to investigate their role in promoting PE.

RETRACTED

## 3. Methodology

### 3.1. IoT-Based PE Framework

This study investigated the physical education program (PEP) grant that is the rotation effect of elementary and intermediate school PE instructors in a quasi-Ohio education system [18]. The main aim of the PEP award for a government-sponsored business is to aid the physical school teachers in providing instructional programs to assure that the understudies enhance their medical status.  Figure 1 shows the IoT-based physical education framework.

The PEP objective of such award is to improve the health of subordinates and implement balanced and enthusiastic physical activities, instead of the usual educating framework that includes the actions of the educational groups. The youngster should be capable of exercising for twenty minutes per day, at least 5 days per week, and strenuous body motions, for a total of 30 minutes per day. At least, three days a week should be devoted to physical activity. The National Association for Sport and Physical Education (NASPE) is an experienced institution dedicated to the advancement of sports and physical education in the USA. The undergraduate students must participate in regular physical activity as quickly as possible in the center [19]. The school teaching days, student medical guidelines, and policies of education account for 7.9%, primary schools, high schools, and only 2.1% of 3.8% [20]. The prize PEP-appropriate central and high school understudies have a variety of functions. Things like data interoperability and reaction advancement are dependent on data from around the world, as well as sophisticated virtual and physical government authorization. Each IoT is made up of a group of European explorers who are responsible for its setup potentials and worldwide organization. It is based on common interoperable interaction principles, with both a virtual and physical basis. It is distinguished by the employment of physical and virtual variables, as well as a smart interface, and it is constantly in collaboration with data organizations to send data to its consumers. IoT, as defined by the GSMA, offers the network's leading edge through lightweight “life-related” device interfaces that completely realized facts [21]. This interconnectedness has a tremendous impact on our lives and works chances. It is also a hint at the link among billions of IoT devices, enhanced healthcare care, transport, efficiency, and energy usage. The agent's only source of power is this connection. Because it is considered a massive information infrastructure, things are true assessment of things information. Fog takes into account new initiatives, connectivity, and a large amount of data. To compute the scores of the principal components of all disciplines in 5G-based sports teaching, every personal information in the preliminary information is inserted into the linear combination equation for all principal components. Average scores indicating the overall quality of the instructor's lessons are absolute indicators relating to students' scores on *m* times of sports tests:

(1) $$\begin{array}{c} \text{Total level}=\frac{T_{s}}{P_{T}}, \end{array}$$

where *T*_*s*_ represents the overall score of times of sports tests and *P*_*T*_ represents the overall count of students engaging in tests. The separation degree employing variance reflecting the online resource sharing classes is

(2) $$\begin{array}{c} {\left(T+S\right)}^{m}=\overset{m}{\underset{k=0}{\sum }}\left(\begin{array}{c} m\\ P \end{array}\right)T_{s}. \end{array}$$

RETRACTED

### 3.2. Model-Based Practice (MBP) of PE

The widely accepted definition of MBP emphasizes the distribution of a single framework. While many investigation studies have looked at how a single framework is delivered and few have looked at hybrid frameworks, some have attempted to relate diverse frameworks in a school's educational program in a meaningful and useful way [22]. To date, no one has empirically explored a broader definition of MBP that incorporates a variety of pedagogical approaches throughout a public school curriculum. Hence, they argue that MBP has stayed connected to Metzler's concept of “model-based” practice instead of the larger umbrella notion of “models-based” practice [23]. For this purpose, they suggest that MBP should be expanded to encompass a wider range of pedagogical models, including (and not restricted to) singular, multi, and mixed models. MBP supports the employment of a range of instructional methods during a PE program [24].

A machine learning-based method of the educational program is made up of a collection of well-chosen primary theme curriculum content, which stands for something meaningful and concentrates on students attaining the aims found as worthwhile of their time and energy [25]. For example, if every student is to successfully meet all of the norms of a physically informed individual by the time they graduate from high school, a multi-model educational program may provide the principle to do so.

MBP is well regarded as a method for achieving considerable PE change. MBP provides for a wider and more in-depth breadth of learning than a single educating framework. Several types of research, such as CL—cooperative learning and TG—tactical games, have looked toward incorporating models and teaching sports for knowledge and sport education [26]. Other research has looked at the relationships between a few concepts [27]. However, no study has looked into the employment of several models across a program [28]. To date, no studies have looked into the MBP described by the following: a model type method to PE might well adopt a diverse of pedagogical methods, each with its number of educational results and orientation of academic results with educational techniques and actual content, and also its own set of non-negotiable advantages in terms of to what educators and students should do to loyally incorporate the prototype [29].

We need the chance to unravel an MBP way of teaching PE that includes several models in the same way that design variables have been examined [30]. We need to specify the educational goals we want for PE (physiological, interpersonal, intellectual, and emotional student learning has been proposed elsewhere), connect them with various models across a program, and then assess and report on the results. We have continually failed to radically reform PE methodology, as suggested, and while MBP is a bright future potential for PE, we need to know a great deal again before we committed to it [31]. If we want to reform the pedagogy of physical education in schools, teachers must be the gatekeepers. It is crucial to comprehend not only the problems and realities that teachers encounter while attempting to execute novel concepts in their classrooms but also how they obtain ownership of those ideas.

RETRACTED

### 3.3. Virtual Reality-Based PE

Virtual reality is being used in a variety of fields, including medicine, media, education, the arts, architecture, tourism, and aviation. The sporting field is no exception. Virtual reality (VR) is used to convey dynamic pictures and a sense of the field during a live sports broadcast. It is also being employed in the sports business, with VR being deployed in the form of a game to allow people to experience sports in reality [32]. Furthermore, because it is situated in a virtual area, which is comparable to reality but regulated, VRT allows for the acquisition of specific technologies. It can be used as the training material to allow physically and mentally challenged persons to participate in sports and rehabilitation because it can be repeated so many times as desired or required. This permits the situation to be set up in a way that is appropriate for impaired people's capacity to use it. This can help to reduce the impact of impairment, enhance the quality of care, encourage people to improve their technology for life, as well as provide great moments [33].

VRT has progressed even faster than the manner of viewing VR utilizing a mask. Virtual avatars now allow for meaningful engagement. It progressed to the point of being a methodology, which may convey the 5 senses [34]. VR technologies, which have been commercially successful in the sports and disability sectors, have a bright future because they allow people with impairments to engage in and enjoy sports, and they may be used to train professional players to enhance sporting event technology. As a result, the goal of this research is to look at examples of VR implementation in individuals with disabilities and sports areas, as well as the tendency of virtual reality subject matter for handicapped people's sports and training experiences, to make sure that VRT shall be used successfully in the future. An example of sports education using virtual reality is displayed in Figure 2.

VR sports that integrate virtual reality methods provide handicapped people with mental and physical limitation option to build up appropriate levels and obtain repeating experiences in a virtual environment that is comparable to reality. Because there are no space or time constraints, it can be used effectively. However, rather than using the latest technology uniformly, it is recommended that virtual reality be used for disabled person's sporting actions in a varied way based on the kind or extent of the damage. Furthermore, when artificial intelligence (AI) is grafting onto the VR method, novel developments are expected not just for nondisabled people's sports and activities, but for disabled people's sports learning and the advancement of technology for elite impaired games practitioners. Because they can study using machine learning when movement data accumulate and because they can identify their difficulties to address by teaching under their own, an era where disabled individuals shall be trained based on the features of their disability [35].

RETRACTED

### 3.4. Internet of Things-Based PE

Through the integration of cost-effective heterogeneous systems with smartphone platforms, the IoT has allowed technology to shift PE to an unregulated, open, or associated world. According to game learning, the IoT opens up a plethora of options for improved education and learning. Minimal communication networks, low bandwidth and storage space, and reduced power computation are only a few of the constraints of IoT equipment. As a result, it is a critical issue for a variety of sensitive applications, including smart homes, which offer secured interaction, power generation, and health information surveillance. Traditional encryption and decryption methods, on the other hand, are unable to make use of the inherent complexity advantage due to their construction and power consumption constraints [36, 37]. In IoT-dependent physical education, quality of services (QoS) refers to a system with higher bandwidth and other system behavior processing, like reliability, error rate, inactivity, and efficacy. Priority regulation over many kinds of network sources is also included under QoS administration. The error rate in the QoS can be computed as

(3) $$\begin{array}{c} \text{Error rate}=Y_{j}-T, \end{array}$$

where *Y* denotes the score on trial *j* and *T* represents the target score. The major aim of quality of service is to offer a lower passivity, dedicated bandwidth, and a preferred network, which comprises regulated vibration and enhanced loss features.

The ball, racquet, and individual body movements are examined for coaching, strategic insights, and projections in sports analysis, which is based on big data. The data in this study are used from expensive luxury cameras mounted in the stadium, and it is a resource of big data analysis on the strong IoT devices in the context. The IoT is a novel breed of web services, which allows physical things to interact with one another over the Internet.

RETRACTED

### 3.5. Artificial Intelligence-Based PE

Artificial intelligence (AI) began to have a profound impact on human existence as science and technology advanced. There has also been a steady increase in the use of AI for sports education [38]. This is a byproduct and an unavoidable outcome of the new exploration mode of PE instruction, as traditional education has no place in the current time. Artificial intelligence may be used in a variety of ways in physical education, including education robots, virtual reality scenarios, educational content, and more. The future of somatic cultivation shall be highly personalized, humanized, and creative under the guidance of AI methodology that has an incalculable effect on physical education and improves the fast emergence of physical education, as shall be seen with the perpetual perfection of scientific and technological standards and the perpetual advancement of the time [39]. In addition to this, the researcher found that IoT-PAMD strategy helps to identify the student's physical health for additional monitoring [40].

## 4. Results and Discussion

In this part, we analyze and compare the various 5G methodologies used for PE. The performance metrics like deployment cost, energy efficiency, and security level are considered for analysis.

### 4.1. Cost Reduction

Connectivity across network connections, comprising capital expenditures (CAPEX) and annual operating costs (OPEX), should be sustained at the least price to create a huge number of computer networks. PE depending on IoT is predicted to provide every customer with relatively low revenue, which will be lower than that of mobile Internet users. This implies a huge number of significant engines for mainstream market applications, as well as conceivable gadgets to make the most out of items, and hence the usage of lower complexity.

The IoT connection is planned to supply every user with very low average revenue per user (ARPU), which will be lower than that of mobile broadband customers. This implies a huge number of significant engines for mass-market utilizations, as well as conceivable gadgets to make the most of things, and hence the usage of lower intricacy. In the context of mobile corporate solutions, production tools, comprising the overall cost of ownership, shall be extremely inexpensive to enable large-scale IoT deployments. Expected summary use cases are assigned to a diverse class with a large permissible delay based on data throughput and update frequency requirements.

### 4.2. Energy Efficiency

Even though the majority of things are battery-powered gadgets that are meant to run without human involvement for a lengthy period, energy efficiency is arguably the most essential element. Hence, PE data security is crucial. Planned and server networking applications in the field of PE must include safety and protection issues. The most crucial element of things is energy efficiency, especially since most things are battery-powered devices that are anticipated to function without human long-term battery usage. Consider a situation in which a fire alarm system sends information directly to the fire department's management. It is necessary to examine such a replacement device that is linked to a clever significant cost component in the time interval between the cells. According to previous studies, most of the amount spent on these goes to interaction device energy. Hardware and software should be designed with energy efficiency in mind.

RETRACTED

### 4.3. Security Level

As a result, the PE statistics should be computed. When it comes to planning and server networking applications in the field of PE, considerations for safety and protection are important. The modern technical explosion has brought safety and privacy concerns to the 5G sphere as well. When we talk about sports in 5G, we have not even touched on this topic. To make 5G-based physical education frameworks work authentically, advancements should be made in this area.  Table 1 shows the comparative analysis of various 5G approaches in the field of PE.

Figure 3 shows the comparative analysis of the cost reduction, energy efficiency, and security level for various 5G technologies employed in physical education. IoT-based PE is better when compared to other techniques.

For PE-related IoT solutions, a pair of wearable Internet of Things will evaluate data collected by complicated intelligent systems, awareness campaigns, and decision-making, moving from a simple architecture to collect, communicate, and visualize through the field, while 5G and IoT technologies have played a significant part in this change. To succeed, we will need a lot of computing power. It is frequently accessible through big data services. The IoT is slowly but steadily changing all aspects of daily life, including education. IoT can also provide additional support to students by predicting academic sustainability or termination. While IoT research is still in its infancy, we must monitor how it develops and manifests its promise over time. We could enhance IoT's potential usage in sports applications and change the character of PE, its visualization, and its repetition by incorporating it into PE.

Virtual reality technology can be utilized to locate unregistered PE pupils during the physical education procedure. Then, via the establishment of neighbor trust, an efficient appraisal of the sports level of sports students could be accomplished. The findings of the study demonstrate that using virtual reality technology in college physical education is one method to change and reinvent the subject. Virtual reality technology will be further advanced in the realm of sports, as evidenced by the preceding analysis. The establishment of a simulation laboratory to move sports to a higher growth direction would be based on the administration of sporting events in the sphere of office automation using information technology. Sports abilities, instruction, and administration can all benefit from virtual reality technology. The most efficient method is to include multimedia technology in sporting events that can boost the efficiency of physical activity. VR sports simulation system is a virtual reality-based training system for professional sports projects. Teachers and learners may constantly develop training activities, acquire the best training impact, and guarantee players' overall fitness by using this elevated training session.

RETRACTED

## 5. Conclusion

The Internet of Things (IoT) development made it possible for technology to communicate physical education by connecting cost-effective heterogeneous devices and digital applications to uncontrolled and accessible environments. In this survey article, we have reviewed the different 5G methodologies utilized for PE. We have analyzed four 5G methodologies which include model-based practice (MBP), virtual reality (VR), the Internet of Things (IoT), and artificial intelligence (AI). The performance measures like cost reduction, energy efficiency, and security level are considered for the comparison analysis. It is observed that IoT-based physical education is efficient in terms of these metrics when compared to the other techniques. This form of the education system was highly favored by students, as evidenced by their desire for practical education with experienced material delivered via smart devices. As a result, to fully utilize 5G, it is necessary to consider boosting a practical, field-oriented educational system. PE needs to be supplemented with more content. A broad curriculum is less vital than improving physical fitness. In the future, more innovations could be developed to improve the performance of the network and the necessity of physical education in today's environment.

## Figures and Tables

**Figure 1:** IoT-based physical education.

**Figure 2:** Sports classroom using virtual reality.

**Figure 3:** Comparison graph for different 5G techniques in physical education.

**Table 1:** Comparative analysis of 5G techniques in physical education.

Author	5G techniques	Cost reduction (%)	Energy efficiency (%)	Security level (%)
Gurvitch et al. [28]	Model-based practice (MBP)	80	80.2	85.9
Kang et al. [36]	Virtual reality (VR)	85	82.5	89.8
Wang et al. [39]	Internet of Things (IoT)	72	94.5	95.6
Wen et al. [38]	Artificial intelligence (AI)	89	88.1	91.5

RETRACTED

## Data Availability

The data underlying the results presented in the study are available within the manuscript.
